# Lipoprotein Ratios: Correlation With Thyroid Profile and Glycated Hemoglobin (HbA1c) Among Diabetes Mellitus Patients

**DOI:** 10.7759/cureus.54191

**Published:** 2024-02-14

**Authors:** Ayan Banerjee, Jagriti LNU, Prabhat LNU, Akash Bansal

**Affiliations:** 1 Biochemistry, All India Institute of Medical Sciences, Patna, Patna, IND; 2 Biochemistry, All India Institute of Medical Sciences, Gorakhpur, Gorakhpur, IND

**Keywords:** hdl-cholesterol, ldl cholesterol, triglyceride, free t3, thyroid-stimulating hormone (tsh), glycated hemoglobin (hba1c)

## Abstract

Introduction: Thyroid disorders and diabetes mellitus are prevalent conditions in the modern era. Moreover, glycated hemoglobin (HbA1c) is the established (prognostic as well as diagnostic) marker for long-term glycemic control, whereas the lipid profile is the marker for cardiovascular risks. The association of hypothyroidism with dyslipidemia is also a well-established fact. The current study explores a correlation between thyroid profile, glycemic status, and various lipoprotein indices.

Objective: To look for an association between thyroid profile, glycemic status, and various lipoprotein indices.

Methodology: The cross-sectional study conducted at AIIMS Gorakhpur included a total of 108 subjects, with 37 normal subjects (Group I) and 71 patients) with T2DM (Type-2 diabetes mellitus) (Group II). Baseline characteristics of the two groups were compared for age, sex, presence of hypertension, fasting blood glucose, and body mass index (BMI). Blood samples were collected from the patients. The sera were analyzed for HbA1c and lipid profile, which included total cholesterol (TC), triglycerides (TG), high-density lipoprotein cholesterol (HDL-C), and low-density lipoprotein cholesterol (LDL-C). Serum samples were also used to estimate the thyroid stimulating hormone (TSH) and triiodothyronine (fT3). The association between thyroid profile, glycemic status, and various lipoprotein indices was calculated.

Statistical analysis:* *Kolmogorov-Smirnov test for normality of the data. Spearmann correlation was used for nonparametric data.

Results: There were significantly higher levels of total cholesterol, triglycerides, and LDL-C levels in T2DM subjects than in non-diabetic subjects. There was also a significant positive correlation observed between TSH and TC among the normal control group (ρ =0.348, P=0.04). Similarly, significant positive correlations were found for TG (ρ =0.354, P=0.04) and LDL-C (ρ =0.431, P=0.03) among non-diabetic subjects. Among patients with T2DM, TSH was significantly correlated positively with TG (ρ =0.530, P=0.006) and LDL-C (ρ =0.443, P=0.03). Similarly, in the same group, among lipid ratios, TG/HDL-C (ρ =0.311, P=0.04) and LDL-C/HDL-C (ρ =0.227, P=0.05) were significantly correlated to TSH. Furthermore, there were significant positive correlations between TSH and HbA1c (ρ =0.301, P=0.04). fT3 was found to have a strong negative correlation with HbA1c among patients with T2DM (ρ =-0.454, P=0.02).

Conclusion: Thyroid disorders exert significant effects on glycemic control and lipid metabolism, which may impact HbA1c levels and lipid profile parameters.

## Introduction

Diabetes mellitus has emerged as an epidemic in India, contributing significantly to premature deaths due to both macro- and micro-vascular complications. The primary factors contributing to the prevalence of type 2 diabetes mellitus (T2DM) include obesity, unhealthy dietary patterns, and fluctuating lifestyles. According to the World Health Organization (WHO), it is projected that by 2025, 134 million Indians will be affected by diabetes mellitus. T2DM primarily manifests through insulin resistance in peripheral organs. In addition to its crucial role in glucose metabolism, insulin also regulates lipid metabolism.

Diabetes mellitus induces alterations in the lipid profile, often resulting in a distinct form of dyslipidemia. The flux of fatty acids to the liver involves the release of fatty acids from adipocytes, a process regulated by insulin. As insulin sensitivity diminishes with the progression towards diabetes mellitus, the natural inhibitory effect on lipid synthesis by the liver and the release of fatty acids from adipocytes are significantly diminished [1].

Characteristic dyslipidemia in diabetic patients is marked by hypertriglyceridemia [2], which stems from increased triglyceride-rich lipoprotein (TRL) synthesis and decreased clearance, both in fasting and non-fasting states. Furthermore, elevated levels of very low-density lipoprotein-cholesterol (VLDL-C) are implicated in hypertriglyceridemia, as VLDL serves as the primary transporter of triglycerides (TG) [3]. Reduced VLDL clearance, decreased hepatic uptake, and elevated postprandial triglyceride-rich chylomicrons contribute to hypertriglyceridemia [2]. High TG levels are directly associated with low levels of high-density lipoprotein cholesterol (HDL-C) [4] and high levels of low-density lipoprotein cholesterol (LDL-C) [5]. Hypertriglyceridemia stimulates the activity of cholesteryl ester transfer protein, leading to the addition of TG to HDL and subsequent catabolism [6]. Additionally, low HDL-C levels, previously attributed to insulin resistance, exacerbate abnormal glucose metabolism [7].

Thyroid disorders, including hypothyroidism and hyperthyroidism, are associated with metabolic disturbances that can impact glycemic control and lipid metabolism. Understanding the correlation between glycated hemoglobin (HbA1c) and lipid profile parameters in patients with thyroid disorders is crucial for comprehensive management and risk stratification in these individuals. Studies have shown that thyroid disorders can influence glycemic control, as reflected by HbA1c levels. Hypothyroidism is commonly associated with dyslipidemia, characterized by elevated total cholesterol (TC), LDL-C, and TG levels, along with decreased HDL-C levels. These lipid profile changes contribute to increased cardiovascular risk in hypothyroid patients.

Limited research has investigated the correlation between HbA1c and lipid profile parameters, specifically in patients with thyroid disorders. Understanding the correlation between HbA1c and lipid profile parameters in patients with thyroid disorders has important clinical implications. Monitoring both HbA1c and lipid profiles regularly can provide a comprehensive metabolic assessment and guide therapeutic interventions in thyroid disorder management.

Our study intends to explore the complex interplay between thyroid function, glycemic control, and lipid metabolism and its implications for cardiovascular risk stratification and management in patients with thyroid disorders.

## Materials and methods

The cross-sectional study included a total of 108 subjects, with 37 normal subjects (group-I) and 71 patients (group-II) with T2DM. The study included individuals visiting the medicine outpatient department (OPD) at AIIMS Gorakhpur. Ethical clearance from the institute’s ethical board had been obtained with reference no. IHEC/AIIMS-GKP/BMR/120/2023 before the initiation of the study. The study was conducted between June 2023 and July 2023.

T2DM patients with a three-year history of disease attending medicine OPD at AIIMS Gorakhpur were enrolled in the study after their bilingual, written, and informed consent.

Patients with type 1 diabetes mellitus, pregnant women, and patients with liver, kidney, or muscle diseases were excluded from the study. Individuals with a previous history of drug treatment for hyperthyroidism, hypothyroidism, serious infections and malignancy, or those taking any drugs known to cause disturbance of lipid metabolism, were also excluded from the study.

A comprehensive examination of subjects included a detailed history relevant general and systemic clinical assessments. Data pertaining to demographics, anthropometrics, clinical details, family history of diabetes, and duration of diabetes were meticulously recorded.

Morning fasting venous blood samples (3 ml) were collected from study participants. Serum samples, obtained by separating whole blood, underwent processing for routine investigations using an automated analyzer, the Olympus AU400, utilizing colorimetric methods. The biochemical parameters assessed for all enrolled subjects were the Lipid profile (including TC, HDL-C, LDL-C, VLDL-C, and TG), HbA1c, thyroid-stimulating hormone (TSH), and free triiodothyronine (fT3). 

HbA1c levels were assessed using micro-column chromatography, while TC and TG levels were determined using an enzymatic method, and HDL-C and LDL-C levels were measured using the direct method. Subsequently, TG/HDL-C, TC/HDL-C, and LDL-C/HDL-C ratios were computed. TSH and fT3 were done using chemiluminescence on the Access 2 Immunoassay System (Beckman Coulter, USA). The normal range of TSH and free T3 considered in the study was 0.27-5.5 µIU/ml and 2.3-4.2 pg/ml, respectively.

Statistical analysis

SPSS Inc. Released 2007. SPSS for Windows, Version 16.0. Chicago, SPSS Inc. was used to code, enter, and analyze all statistical data. Descriptive statistical methods were employed to access the data, and the Kolmogorov-Smirnov test was used to determine if the parameters followed a normal distribution. Continuous variables were presented as the mean and standard deviation (SD). Pearson’s correlation and Spearman correlation studies were done for parametric data and non-parametric data, respectively. Statistical significance was defined as a p-value ≤ 0.05 after analyzing the findings and 95% confidence intervals (CI).

## Results

The study enrolled a total of 108 subjects, with group-I comprising 37 normal (control) subjects with HbA1c <6.5 and group-II comprising 71 subjects with T2DM (HbA1c ≥6.5). Table 1 reflects the various parameters of the lipid profile and thyroid profile of two groups of subjects. The two groups were comparable, with no significant difference in terms of age, sex, or body mass index (BMI) (Table 1). However, only 11% and 5% of subjects in group-I had metabolic syndrome and hypertension, respectively (Table 1). In addition, a significantly higher number of subjects, namely 37% and 31%, had metabolic syndrome and hypertension, respectively, in group-II (Table 1). Similarly, there were significantly higher levels of TC, TG, and LDL-C in group-II in comparison to group-I (Table 1). Similarly, there were significantly higher levels of TSH in patients with T2DM in comparison to normal subjects (Table 1). However, fT3 levels were significantly lower among diabetic subjects than in normal subjects (Table 1).

**Table 1:** Baseline characteristics of study subjects based on HbA1c levels Difference between groups (p≤0.05=significant*, p≤0.001= highly significant**) BMI: Body mass index; TG: Triglyceride, HDL-C: High-density lipoprotein cholesterol, LDL: Low-density lipoprotein cholesterol, TSH: Thyroid stimulating hormone, fT3: free triiodothyronine

Parameters	Group-I (HbA1c <6.5): N=37	Group-II (HbA1c ≥6.5); N=71	P-value
Age (years)	46.14±6.15	48.74±7.81	0.08
Sex (Male:Female)	22 (59%):15 (41%)	50 (70%):21 (30%)	p>0.05
BMI (Kg/m^2^)	31.14±3.11	32.13±4.02	0.194
Fasting blood glucose (mg/dl) *	92.1±10.3	160.2±52.3	0.001
With Hypertension*	4 (11%)	22 (31%)	0.001
With Metabolic syndrome*	2 (5%)	26 (37%)	0.001
Total Cholesterol* (mg/dl)	160±39	181±56	0.04
TG (mg/dl) *	145±26	163±51	0.05
HDL-C(mg/dl)	39±14	36±9	0.18
LDL-C(mg/dl) *	96±38	121±52	0.01
TSH(µIU/ml) **	3.5±1.4	5.5±1.2	0.001
fT3(pg/ml) *	3.1±0.7	2.1±0.8	0.04

There was also a significant positive correlation observed between TSH and TC among the normal control group (Table 2) (ρ =0.348, P=0.04). Similarly, significant positive correlations were found for triglycerides (ρ =0.354, P=0.04) and LDL-C (ρ =0.431, P=0.03) (Table 2). Conversely, HDL-C was negatively correlated to TSH, but was non-significant for control group subjects (Table 2). Among lipid ratios, TG/HDL-C (ρ =0.342, P=0.05) and total cholesterol/HDL-C (ρ =0.341, P=0.05) were significantly positively correlated to TSH levels. HbA1c, though positively correlated to TSH, was non-significant (ρ =0.213, P=0.19) (Table 2).

**Table 2:** Correlation of lipid indices and HbA1c with TSH (HbA1c <6.5) Correlation is significant at the 0.05 (2-tailed) level * TG: Triglyceride, HDL-C: High density lipoprotein cholesterol, LDL-C: Low-density lipoprotein cholesterol, TSH: Thyroid stimulating hormone, HbA1c: Glycated hemoglobin

Parameters	Spearman Correlation	
N=37	Spearman correlation coefficient (ρ)	P-value
Total Cholesterol	0.348*	0.04
TG	0.354*	0.04
HDL-C	-0.105	0.57
LDL-C	0.431*	0.03
TG/HDL-C	0.342*	0.05
Total Cholesterol/HDL-C	0.341*	0.05
Non-HDL-C/HDL-C	0.24	0.19
LDL-C/HDL-C	0.241	0.19
HbA1c	0.213	0.19

Among patients with T2DM, TSH was significantly correlated positively with triglycerides (ρ =0.530, P=0.006) and LDL-C (ρ =0.443, P=0.03) (Table 3). Similarly, among lipid ratios, TG/HDL-C (ρ =0.311, P=0.04) and LDL-C/HDL-C (ρ =0.227, P=0.05) were significantly correlated to TSH. Furthermore, there were significant positive correlations between TSH and HbA1c (ρ =0.301, P=0.04) (Table 3).

**Table 3:** Correlation of lipid indices and HbA1c with TSH (HbA1c ≥6.5) Correlation is significant at the 0.05 (2-tailed) level * TG: Triglyceride, HDL-C: High density lipoprotein cholesterol, LDL-C: Low-density lipoprotein cholesterol, TSH: Thyroid stimulating hormone, HbA1C: Glycated hemoglobin

Parameters	Spearman Correlation	
N=71	Spearman correlation coefficient (ρ)	P-value
Total Cholesterol	0.205	0.07
TG	0.530*	0.006
HDL-C	-0.192	0.12
LDL-C	0.443*	0.03
TG/HDL-C	0.311*	0.04
Total Cholesterol/HDL-C	-0.195	0.12
Non-HDL-C/HDL-C	-0.195	0.12
LDL-C/HDL-C	0.227*	0.05
HbA1c	0.301*	0.04

Similarly, correlation studies were done with various parameters of the lipid profile and their ratios in comparison to fT4 but were non-significant. However, fT4 was found to have a strong negative correlation with HbA1c among patients with T2DM (ρ =-0.454, P=0.02) (Table 4). Though, similar correlations were not found among normal subjects with HbA1c <6.5 (Table 4).

**Table 4:** Correlation between fT3 and HbA1c Correlation is significant at the 0.05 (2-tailed) level * HbA1C: Glycated hemoglobin, fT3: free T3

Parameters	Spearman Correlation	
	Spearman correlation coefficient (ρ)	P-value
HbA1c <6.5(N=37)	0.264	0.14
HbA1c ≥6.5(N=71)	-0.454*	0.02

## Discussion

Diabetes, an endocrine metabolic disorder, poses a significant public health threat and stands as a primary cause of morbidity and mortality globally [8]. Thyroid dysfunction and T2DM are prevalent endocrinal disorders encountered in routine clinical practice, yet their underlying mechanisms remain incompletely understood [9]. An association between diabetes and thyroid dysfunction exists, bearing notable clinical implications [10-12]. Thyroid hormones play a crucial role in regulating lipid metabolism [2,13], and thyroid dysfunction is often linked with dyslipidemia [14], whereas T2DM is characterized by abnormal blood lipid profiles [15]. Although numerous studies have examined the relationship between thyroid hormones and lipid abnormalities, relatively few have specifically investigated this association in patients with T2DM [16].

In our investigation, T2DM patients exhibited higher serum levels of TC, LDL-C, and TG compared to non-diabetic subjects. Numerous studies have explored the relationship between HbA1c and lipid profile parameters to understand their interconnectedness within metabolic disorders. For instance, a study by Zhe et al. [17] revealed a positive correlation between HbA1c levels and TC, as well as LDL-C. Additionally, HbA1c has been directly associated with cardiovascular risks [18]. In a cross-sectional retrospective analysis conducted by A. Y. Sharahili et al. [19], higher HbA1c levels were significantly linked with unfavorable lipid profiles characterized by elevated LDL-C and TG levels, along with reduced HDL-C levels, independent of other metabolic risk factors.

In our study, T2DM patients exhibited significantly lower serum levels of fT4, while the serum level of TSH was notably higher compared to non-diabetic subjects. These findings are consistent with previous reports [20-23]. However, Anveetha et al. [24] reported increased serum levels of TSH and fasting blood sugar (FBS) among 30 patients with T2DM, along with lower levels of T3 and T4 compared to healthy control subjects. Diabetes-induced alterations in the hypothalamic-pituitary-thyroid axis lead to reduced synthesis and release of thyroid-releasing hormone (TRH), limiting iodide uptake by the thyroid gland and consequently reducing T3 and T4 production [25,26].

Furthermore, our study revealed a positive association between low thyroid function and lipid dysregulation in T2DM patients, with a significant positive relationship observed between TSH and TG, LDL-C, and TC, along with an insignificant negative correlation between TSH and HDL-C among normal subjects. Similarly, among patients with T2DM, TSH was significantly correlated positively with TG (ρ =0.530, P=0.006) and LDL-C (ρ =0.443, P=0.03). Our findings are in contrast with reports by Chubb et al. [27] and Zhang et al. [28], who demonstrated a significant negative correlation between serum HDL-C and TSH in T2DM patients and non-diabetic subjects. Similar findings have been described by several researchers [29,30].

However, Giandalia et al. [31] and Triolo et al. [32] reported a significant association between TSH and high triglycerides in T2DM patients, which may be related to visceral obesity and an increased susceptibility to atherosclerosis in T2DM. Moreover, the positive correlation between TSH and TG, TC, and LDL-C may be attributed to the activation of autoimmunity involved in lipoprotein production [33].

Our study found that fT3 had a strong negative correlation with HbA1c among patients with T2DM (ρ =-0.454, P=0.02). Similar findings were reported by Udenze et al. in patients with metabolic syndrome in Lagos, Nigeria [34]. This decline in T3 levels could be attributed to the prolonged effects of hyperglycemia on the peripheral deiodination of T4 to T3 and/or the attenuation of nocturnal peaks in TRH secretion due to chronic hyperglycemia in T2DM patients [35]. Poorly managed diabetes has been associated with a "low T3 state," characterized by reduced serum total and fT3 levels [35].

Furthermore, among the majority of T2DM patients with hypothyroidism in this study, there was an inverse correlation between HbA1c and serum fT3 levels and a positive correlation between HbA1c and TSH levels. This relationship may be attributed to the impact of chronic hyperglycemia observed in T2DM on the peripheral conversion of T4 to T3. Similar findings were reported by Bazrafshan et al. in Gorgan, Iran (36), who observed a positive correlation between HbA1c and TSH levels in T2DM patients. Consistent results were also reported by Asmabi et al., who studied 100 patients with diabetes.

Study limitations: The study had a small sample size. A large-scale study needs to be conducted with a wider range of populations for generalized results. Moreover, the study was conducted at a single center, which was another limitation. A similar multicentric study can be done to address ethnic variability.

## Conclusions

Thyroid disorders exert significant effects on glycemic control and lipid metabolism, which may impact HbA1c levels and lipid profile parameters. The current study suggests significant correlations between TSH and parameters of the lipid profile among normal subjects and patients with T2DM. Furthermore, TSH was positively correlated with HbA1c among patients with T2DM. Given that early signs and symptoms of thyroid disorders often go unnoticed, undiagnosed cases could detrimentally impact diabetes management and its associated complications. Thus, routine screening of thyroid profiles in diabetic patients is recommended and deemed advantageous to enhance the quality of life, diminish morbidity rates, and mitigate complications.

While existing evidence suggests associations between thyroid function, HbA1c, and lipid profile, further research is needed to clarify these relationships and optimize metabolic management in patients with thyroid disorders.

## References

[1] (2024). Jama Cardio: The engima of glucose and lipid metabolism. http://10.1001/jamacardio.2016.0183.

[2] Wu L, Parhofer KG (2014). Diabetic dyslipidemia. Metabolism.

[3] Saleh J, Sniderman AD, Cianflone K (1999). Regulation of plasma fatty acid metabolism. Clin Chim Acta Int J Clin Chem.

[4] Quispe R, Manalac RJ, Faridi KF (2015). Relationship of the triglyceride to high-density lipoprotein cholesterol (TG/HDL-C) ratio to the remainder of the lipid profile: The very large database of lipids-4 (VLDL-4) study. Atherosclerosis.

[5] Sniderman AD, Couture P, Martin SS (2018). Hypertriglyceridemia and cardiovascular risk: a cautionary note about metabolic confounding. J Lipid Res.

[6] Guérin M, Le Goff W, Lassel TS, Van Tol A, Steiner G, Chapman MJ (2001). Atherogenic role of elevated CE transfer from HDL to VLDL(1) and dense LDL in type 2 diabetes : impact of the degree of triglyceridemia. Arterioscler Thromb Vasc Biol.

[7] Drew BG, Rye KA, Duffy SJ, Barter P, Kingwell BA (2012). The emerging role of HDL in glucose metabolism. Nat Rev Endocrinol.

[8] Bulum T, Kolarić B, Duvnjak L (2012). Insulin sensitivity modifies the relationship between thyroid function and lipid profile in euthyroid type 1 diabetic patients. Endocrine.

[9] Peppa M, Koliaki C, Nikolopoulos P, Raptis SA (2010). Skeletal muscle insulin resistance in endocrine disease. J Biomed Biotechnol.

[10] Liu H, Peng D (2022). Update on dyslipidemia in hypothyroidism: the mechanism of dyslipidemia in hypothyroidism. Endocr Connect.

[11] Raghuwanshi P, Rajput D, Ratre B, Jain R, Patel N, Jain S (2014). Evaluation of thyroid dysfunction among type 2 diabetic patients. Asian J Med Sci.

[12] Duntas LH, Orgiazzi J, Brabant G (2011). The interface between thyroid and diabetes mellitus. Clin Endocrinol (Oxf).

[13] Roos A, Bakker SJ, Links TP, Gans RO, Wolffenbuttel BH (2007). Thyroid function is associated with components of the metabolic syndrome in euthyroid subjects. J Clin Endocrinol Metab.

[14] Lambadiari V, Mitrou P, Maratou E, Raptis AE, Tountas N, Raptis SA, Dimitriadis G (2011). Thyroid hormones are positively associated with insulin resistance early in the development of type 2 diabetes. Endocrine.

[15] Strollo F, Carucci I, Morè M, Marico G, Strollo G, Masini MA, Gentile S (2012). Free triiodothyronine and cholesterol levels in euthyroid elderly T2DM patients. Int J Endocrinol.

[16] Papadopoulou AM, Bakogiannis N, Skrapari I, Moris D, Bakoyiannis C (2020). Thyroid dysfunction and atherosclerosis: A systematic review. In Vivo.

[17] Yan Z, Liu Y, Huang H (2012). Association of glycosylated hemoglobin level with lipid ratio and individual lipids in type 2 diabetic patients. Asian Pac J Trop Med.

[18] Kayali Y, Ozder A (2021). Glycosylated hemoglobin A1c predicts coronary artery disease in non-diabetic patients. J Clin Lab Anal.

[19] Sharahili AY, Mir SA, ALosari S (2023). Correlation of HbA1c level with lipid profile in type 2 diabetes mellitus patients visiting a primary healthcare center in Jeddah City, Saudi Arabia: a retrospective cross-sectional study. Diseases.

[20] Mehalingam V, Sahoo J, Bobby Z, Vinod KV (2020). Thyroid dysfunction in patients with type 2 diabetes mellitus and its association with diabetic complications. J Family Med Prim Care.

[21] Saeed WM, Elrahman SFA, Abdrabo AA (2016). Evaluation of thyroid function test in Sudanese patients with type 2 diabetes mellitus. Sema Sch.

[22] Witting V, Bergis D, Sadet D, Badenhoop K (2014). Thyroid disease in insulin-treated patients with type 2 diabetes: a retrospective study. Thyroid Res.

[23] Demitrost L, Ranabir S (2012). Thyroid dysfunction in type 2 diabetes mellitus: A retrospective study. Indian J Endocrinol Metab.

[24] Suzuki Y, Nanno M, Gemma R, Tanaka I, Taminato T, Yoshimi T (1994). [The mechanism of thyroid hormone abnormalities in patients with diabetes mellitus]. Nihon Naibunpi Gakkai Zasshi.

[25] Chubb SA, Davis WA, Davis TM (2005). Interactions among thyroid function, insulin sensitivity, and serum lipid concentrations: the Fremantle diabetes study. J Clin Endocrinol Metab.

[26] Zhang Y, Lu P, Zhang L, Xiao X (2015). Association between lipids profile and thyroid parameters in euthyroid diabetic subjects: a cross-sectional study. BMC Endocr Disord.

[27] Asvold BO, Vatten LJ, Nilsen TI, Bjøro T (2007). The association between TSH within the reference range and serum lipid concentrations in a population-based study. The HUNT Study. Eur J Endocrinol.

[28] Rizos CV, Elisaf MS, Liberopoulos EN (2011). Effects of thyroid dysfunction on lipid profile. Open Cardiovasc Med J.

[29] Witte T, Ittermann T, Thamm M, Riblet NB, Völzke H (2015). Association between serum thyroid-stimulating hormone levels and serum lipids in children and adolescents: a population-based study of german youth. J Clin Endocrinol Metab.

[30] Giandalia A, Russo GT, Romeo EL (2014). Influence of high-normal serum TSH levels on major cardiovascular risk factors and Visceral Adiposity Index in euthyroid type 2 diabetic subjects. Endocrine.

[31] van Tienhoven-Wind LJ, Dullaart RP (2015). Low-normal thyroid function and novel cardiometabolic biomarkers. Nutrients.

[32] Bakker O, Hudig F, Meijssen S, Wiersinga WM (1998). Effects of triiodothyronine and amiodarone on the promoter of the human LDL receptor gene. Biochem Biophys Res Commun.

[33] Lopez D, Abisambra Socarrás JF, Bedi M, Ness GC (2007). Activation of the hepatic LDL receptor promoter by thyroid hormone. Biochim Biophys Acta.

[34] Hage M, Zantout MS, Azar ST (2011). Thyroid disorders and diabetes mellitus. J Thyroid Res.

[35] H. R.Bazrafshan (M.D), M. A.Ramezani (M.D), A. Salehei (M.D) (2000). Thyroid dysfunction and its relation with diabetes mellitus (NIDDM). J Gorgan Univ Med Sci.

